# Study on the Effect of MRI in the Diagnosis of Benign and Malignant Thoracic Tumors

**DOI:** 10.1155/2021/3265561

**Published:** 2021-12-20

**Authors:** Yan Li, Yangli Sui, Mingyan Chi, Jie Zhang, Lin Guo

**Affiliations:** ^1^Department of Health Examination, Penglai Hospital of Traditional Chinese Medicine, Yantai City, Yantai, Shandong 265600, China; ^2^Department of Imaging, Penglai Hospital of Traditional Chinese Medicine, Yantai City, Yantai, Shandong 265600, China; ^3^Department of Ultrasound, Penglai Hospital of Traditional Chinese Medicine, Yantai City, Yantai, Shandong 265600, China; ^4^Department of Medical Records, Penglai Hospital of Traditional Chinese Medicine, Yantai City, Yantai, Shandong 265600, China; ^5^Department of Physical Examination of Traditional Chinese Medicine, Yantai Penglai Hospital of Traditional Chinese Medicine, Yantai City, Yantai, Shandong 265600, China

## Abstract

In order to investigate the effectiveness and accuracy of magnetic resonance imaging (MRI) in the diagnosis of benign and malignant thoracic tumors, the research retrospectively selected 80 patients with thoracic tumors admitted from May 2019 to May 2020 as the study subject and all patients were underwent MRI detection. Using pathological diagnostic results as the gold standard, the research analyzed the detection of benign and malignant thoracic tumors by MRI, as well as the diagnostic sensitivity and specificity. After pathological diagnosis, there were 35 malignant tumors and 45 benign tumors. 41 cases of malignant tumors and 39 cases of benign tumors were diagnosed by MRI, with a diagnostic sensitivity of 80.00%, a diagnostic specificity of 71.11%, and a diagnostic compliance rate of 75.00%. In the MRI diagnosis of tumors in different parts of the chest, the diagnostic sensitivity for lung tumors, mediastinal tumors, chest wall tumors, and esophageal tumors was 83.33%, 71.43%, 83.33%, 75.00%, and 87.50%, respectively, and the specificity was 66.67%, 77.78%, 57.14%, 50.00%, and 91.67% according to and breast tumors, respectively. And the accuracy was 73.33%, 75.00%, 69.23, 62.50%, and 90.00%, respectively, with the highest diagnostic sensitivity, specificity, and accuracy for breast tumors. MRI has a good effect on the diagnosis of benign and malignant thoracic tumors and has a high diagnostic value, which is helpful to identify the location, nature, source, and lesion scope of the tumor. It is safe and worthy of promotion.

## 1. Introduction

There are many different types of chest tumors. Anatomically, thoracic tumors are mainly divided into several categories: lung tumors, mediastinal tumors, chest wall tumors, esophageal tumors, and mammary gland tumor. The pathogenesis and physiological type of the disease are relatively complex, especially malignant tumor diseases such as lung cancer, which are highly metastatic, and the morbidity and mortality rates have been increasing year by year in recent years [1, 2]. Pathologically, there is also a difference between benign and malignant. The diagnosis of benign and malignant thoracic tumors is crucial to the choice of treatment and assessment of prognosis. Therefore, the differentiation of benign and malignant thoracic tumors becomes the key and difficult part of clinical treatment. Therefore, early detection of thoracic tumors and accurate determination of tumor nature to achieve early diagnosis and treatment of tumors are especially important for the life and health of patients. The deep thoracic soft tissue, muscle, and bone tissues of the human body are complex, the tumor origin and pathological types involved are various, and some patients do not have specific symptoms in the early stage of the tumor, so the misdiagnosis rate of chest wall tumors based on medical history, symptoms, physical examination, and the nature of the mass is high [3]. CT of the chest is the first choice for imaging of chest diseases, but some solid chest masses have no enhancement on CT enhancement, while some cystic masses have increased CT values in the cystic cavity due to internal bleeding and infection, which can easily lead to misdiagnosis and thus delay treatment [4]. MRI is a new medical imaging technique with high diagnostic performance for parenchymal organs such as brain, thyroid, liver, gallbladder, spleen, kidney, pancreas, adrenal gland, uterus, ovary, prostate, and heart and large blood vessels [5]. Compared with other auxiliary examinations such as X-ray and CT, MRI has the advantages of multiple imaging parameters, fast scanning speed, high tissue resolution, and clearer images, which can not only detect tumors, cerebral infarction, cerebral hemorrhage, cerebral abscess, cerebral cysticercosis, and congenital cerebrovascular malformations at an early stage but also determine the types and causes of hydrocephalus, and thus, MRI is more widely used in the screening and diagnosis of brain diseases [2]. At the same time, MRI does not expose patients to any ionizing radiation and can help distinguish pulmonary malignancies, certain sarcoidosis, and pulmonary malignancies by the size of fatty grains. Routine MR examination sequences in the chest include T2W and its fat suppression sequence and TIW and its chemical shift imaging sequence, which can show breast, mediastinal and lung masses, and surrounding structures, including location, size, morphology, tumor-lung interface, and contour [6, 7]. Based on this, this study used MRI for benign and malignant diagnosis of lung cancer, breast tumors, and other chest tumors as a way to broaden the prospects of MRI applications and also to explore new ideas for early diagnosis of chest diseases and to improve the diagnostic efficacy of chest malignancies.

## 2. Method

### 2.1. Inclusion Criteria and Exclusion Criteria

In this study, patients with thoracic tumor were retrospectively selected as subjects, and all patients underwent MRI detection. Inclusion criteria: ① all patients with occupying renal lesions according to imaging and clinical diagnosis and pathological diagnosis by surgery or diagnostic puncture in our hospital, and their medical records were complete and correct; ② all patients voluntarily signed informed consent form. Exclusion criteria: ①combined with serious chest diseases or other organ function damage; ② combined with infectious diseases; ③ patients with metal implants in the body, such as cardiac coronary stents and metal internal fixation stents; ④ patients with claustrophobia; and ⑤ various causes of image motion artifacts or heavy magnetic sensitivity artifacts that significantly affect the reading and measurement of lesions.

The study was approved by the Medical Ethics Committee (No. 201922), and the protocol was developed in accordance with the relevant requirements of the World Medical Association Declaration of Helsinki.

### 2.2. Diagnosis Method

In order to reduce artifacts due to respiratory motion, all patients underwent breathing training before MRI scanning, holding their breath at the end of inspiration after a deep breath. All patients underwent MRI scans with a Siemens Avanto 1.5T MRI scanner (Simenns) for MRI scans of the patient's chest with conventional sagittal sequences (T1WI, transaxial T1WI, T2WI, FLAIR, and DWI sequences) and coronal T2WI, diffusion-weighted imaging with a 16-channel cephalometric phased-array coil, and enhanced scans by selecting 0.01 mmol/kg gadopentetate glucosamine [7]. T1WI parameters are as follows: repetition time (TR)/echo time (TE) = 2500/30 ms, scanning field of view (FOV) = 23 cm × 23 cm, layer thickness = 6 mm, layer spacing 20%, matrix = 256 × 256, and inversion angle = 70°; T2WI parameters are as follows: TR = 1580/72 ms, FOV = 22 cm × 22 cm, layer thickness = 6 mm, and matrix = 256 × 256; DWI parameters are as follows: TR = 6800/70 ms, TE = 84/85 Efms, FOV = 22 cm × 22 cm, layer thickness = 6 mm, *b* = 1000 s/mm^2^, and matrix = 256 × 256. The MRI scanning images are uploaded to the scanner processing station and reviewed by three experienced imaging physicians, who focus on the location and morphology of the lesion from the MRI scan routine sequence, measure the lesion area in the high signal area on the DWI image, analyze the benign and malignant nature of the chest tumor, and make a final diagnosis after discussion of the images that are questionable. This study adopted image blinding reading, and the imaging physicians were unaware of the pathological results. The patient's surgical pathology or puncture biopsy results are used as the “gold standard.”

### 2.3. Observed Indicators

The pathological diagnostic results were recorded. The number of benign and malignant tumor cases was recorded, and their imaging characteristics were analyzed according to the MRI scan results and diagnostic results. At the same time, the diagnostic efficacy of MRI for different chest tumors, including sensitivity, specificity, and accuracy, was also analyzed by using the pathological diagnostic results as the gold standard.

Diagnostic sensitivity = number of true − positive cases/(number of true − positive cases + number of false − negative cases)∗100%, diagnostic specificity = number of true − negative cases/(number of true − negative cases + number of false − positive cases)∗100%, and diagnostic compliance rate = (number of true − positive cases + number of true − negative cases)/total number of cases∗100% [8].

### 2.4. Statistical Methods

The data obtained were analyzed by the SPSS 22.0 statistical software, and the measurement data were expressed by (), and the *t*-test was used for the comparison between groups of measurement data conforming to normal distribution; the count data were expressed by *n* (%), and the *χ*^2^ test was performed between groups, and the Kappa test was used for consistency (Kappa > 0.75 indicates excellent consistency, 0.4-0.75 indicates ideal consistency, and <0.4 indicated poor consistency). *P* < 0.05 indicated that the difference was statistically significant.

## 3. Result

### 3.1. General Information

This study retrospectively collected 80 patients admitted to our hospital from May 2019 to May 2020, including 45 male patients and 35 female patients. The age ranged from 23 to 78 years old, with a mean age of 52.57 ± 7.48 years old. The mean age of patients in the benign tumor group was 41.32 ± 9.68 years old, and the mean age of patients in the malignant tumor group was 54.82 ± 6.53 years old, and the age of patients in the benign tumor group was less than that of patients in the malignant tumor group, but the difference was not statistically significant (*P* > 0.05). The benign tumor group included 21 male patients and 18 female patients, and the malignant tumor group included 24 male patients and 17 female patients, and there was no statistically significant difference in gender between the two groups (*P* > 0.05; Table 1).

### 3.2. The Diagnostic Value of MRI for Benign and Malignant Thoracic Tumors

According to MRI diagnosis, 80 patients contained 41 (51.25%) malignant tumors and 39 (48.75%) benign tumors. By pathological diagnosis, 35 cases (42.75%) of malignant tumors and 45 cases (56.25%) of benign tumors were included. The diagnostic sensitivity was 80.00%, the diagnostic specificity was 71.11%, and the diagnostic compliance rate was 75.00%. There was no significant difference between MRI diagnosis of benign and malignant tumor of chest and pathological results (*P* > 0.05). The consistency between MRI diagnosis and its diagnosis of benign and malignant thoracic tumors was more ideal (Kappa = 50.16%) with reference to the pathological diagnosis results of surgery or puncture biopsy.

Details are shown in Table 2.

### 3.3. Analysis of the Detection Results of Benign and Malignant Tumors in Different Parts of the Chest

The site of the tumor helps to determine the source of the tumor. The MRI detection rate for chest tumors in different site was 100.00%, and the diagnostic sensitivity of lung tumor, mediastinal tumor, chest wall tumor, esophageal tumor, and breast tumor is 83.33%, 71.43%, 83.33%, 75.00%, and 87.50%, respectively. The specificity was 66.67%, 77.78%, 57.14%, 50.00%, and 91.67%, respectively, and the accuracy was 73.33%, 75.00%, 69.23%, 62.50%, and 90.00%, respectively. The sensitivity, specificity, and accuracy of breast tumor were the highest. Details are shown in Tables 3 and 4 and Figures 1 and 2.

### 3.4. Analysis of MRI Imaging Features of Benign and Malignant Thoracic Tumors

The morphology, boundary, and lymph node metastasis of chest tumor are the most visual reflection of its biological behavior, which helps to judge the benign and malignant tumors. Irregular tumor morphology often indicates that the tumor has the characteristics of fast growth and high aggressiveness. Therefore, this study further analyzed the MRI imaging characteristics of different chest tumors and found that the MRI performance of benign and malignant tumors had significant differences in morphology, boundary, invasion and lymph node metastasis, etc., with *P* < 0.05, which was statistically significant (Table 5).

## 4. Discussion

As living environment, living habits, diet, and other factors closely related to human health continue to change, rapid diagnosis and timely treatment of thoracic tumor diseases have attracted wide attention under the background of increasing incidence of thoracic tumor diseases, deepening attention to health, and continuous development of medical technology and medical services [1, 2]. Chest tumors include lung tumors, mediastinal tumors, chest wall tumors, esophageal tumors, and breast tumors, with intricate pathologic mechanisms and prone to metastasis or other complications, leading to multiple organ dysfunction and seriously threatening patients' lives [9]. Therefore, it is of great significance for patients and their families to continuously explore new diagnostic methods for thoracic tumors, improve diagnostic accuracy and diagnostic efficiency, and take timely treatment measures for patients.

X-rays and CT are commonly used for the diagnosis of chest diseases. CT can present three-dimensional images as a way to analyze the relationship between tumor tissues and their surroundings; X-ray imaging can diagnose the origin of the tumor, such as chest wall tumor bone or from soft tissue [10] in X-ray and benign soft tissue tumors image as round or oval shadows of masses with uniform distribution and clearer and more definite margins in local areas. In contrast, malignant tumors exhibit lamellar shadows with curved, lobulated edges [8, 11]. However, at the same time, X-rays and CT are essential images of the spatial distribution of tissue absorption of X-rays. When the focal tissue of the lesion absorbs the same coefficient of X-rays as the adjacent normal tissue in the early stage of development, it is very easy to misdiagnose and miss the diagnosis by using X-ray techniques. However, X-ray and CT diagnosis after tissue lesions have reached a certain degree, or lesions have formed may delay the optimal treatment opportunity [10].

Compared with X-rays and CT, MRI has been used later in clinical medicine and mainly uses static and radiofrequency magnetic fields to form clear images of human tissues with high contrast, which neither requires the use of contrast agents nor is affected by electronic radiation, and is now mostly used in clinical practice to diagnose brain tissue lesions and neurological disorders [12]. In this study, MRI was used to diagnose thoracic tumors as a way to broaden the prospects of MRI application and to explore new ideas for early diagnosis of thoracic diseases. The results showed that among 80 patients with chest tumors, MRI diagnosed 35 malignant tumors and 45 benign tumors. Using pathological diagnosis as the gold standard, the diagnostic sensitivity of MRI was 80.00%, the diagnostic specificity was 71.11%, the diagnostic compliance rate was 75.00%, and the accuracy rate of diagnosing different types of chest tumors using a single MRI technique was 100.00%. Kappa values indicate that MRI diagnosis is in better ideal consistency with its diagnosis of benign and malignant thoracic tumors. This indicates that MRI has a high diagnostic efficacy for the orientation and type of thoracic tumor lesions located. The reason for this is that MRI can use different instrument parameters to analyze the distribution size, range, and orientation of the lesion tissue from the conventional sagittal sequence (T1WI, transverse T1WI, T2WI, FLAIR, and DWI sequence) and coronal position at multiple levels and angles, as well as the change of tissue density and the identification of tumor properties [13]. Diffusion-weighted imaging (DWI) can reflect the Brownian motion of tissue water molecules. Due to different tissue structures, water molecules do not move randomly, so they are limited by collisions with cells in tissues, hydrophobic membranes, and intracellular macromolecules. DWI technology can be sensitive to detect changes in the diffusion of water molecules at the cellular level. In recent years, DWI imaging parameters have become increasingly standardized and image quality has been significantly improved, which is of great value in differentiating benign and malignant chest nodules [14, 15].

In this study, MRI had the highest diagnostic sensitivity, specificity, and accuracy for breast tumors, which were 87.50%, 91.67%, and 90.00%, respectively. Breast cancer occupies the first place among female malignant tumor diseases in China, and due to the excessive amount of adipose tissue and radiation, X-rays and CT multiple scans are detrimental to patients' health. T2 signals were based on the principle of NUCLEAR magnetic resonance, thus reflecting the relationship of human tissue structure. At the same time, MRI has a high resolution of soft tissue, and the special control front ring for breast can be used to naturally hang both mammary glands to reduce the interference of external factors, improve image quality, and increase the specificity and sensitivity of MRI diagnosis of breast cancer [13, 16]. Breast cancer has a burr sign due to its tendency to invade surrounding tissues and thus has unclear borders with them. And MRI can effectively reflect the changes of burrs in breast cancer patients, thus effectively improving the diagnostic efficiency [17]. In general, benign mammary mass is mostly round or circular in shape and has well-defined borders with lobulated or smooth edges. In contrast, the MRI sign of breast cancer lies in the lack of clear demarcation between it and the mass and the surrounding tissues or the irregular, burr-like, or jagged borders of the mass. It also contains a heterogeneous internal signal and may be accompanied by local skin thickening, nipple depression, and axillary lymph node enlargement [16, 18].

Besides, MRI still has some limitations and still needs to be combined with other diagnostic measures for joint diagnosis. For example, if there is only a small amount and subtle degree of calcification appears in the tumor tissue in the early stage, the diagnostic sensitivity of MRI is not high, and it still needs to be combined with X-ray for diagnosis [19, 20]. Moreover, the thoracic tumor tissue is complex, and when benign and malignant tumors exist at the same time, the overlapping effects will interfere with MRI diagnosis, and other three-dimensional effects are also needed to cooperate with multiangle and multilevel collection of impact information [12]. In addition, the price of clinical MRI diagnosis is higher compared with the routinely used X-ray and CT, and it is also difficult for comprehensive popularization [21].

In conclusion, MRI is more effective and safer for diagnosing benign and malignant thoracic tumors and can be used to determine the tumor site of chest diseases in the early stage and combined with other examinations to further improve the diagnosis of tumor information such as tumor nature and regional size. This study also has the following shortcomings: this study is a single-center, small-sample retrospective study, which may be biased and needs to be further discussed in a large-sample multicenter.

## Figures and Tables

**Figure 1:** Malignant tumor of the right side of the lung in the chest.

**Figure 2:** Adrenal metastasis of lung tumor.

**Table 1:** Comparison of patient general information.

Group	Age (yeas old)	Male/female (unit)
Benign tumor	41.32 ± 9.68	21/18
Malignant tumor	54.82 ± 6.53	24/17
*F*/*χ*^2^ value	13.2	15.30
*P* value	0.82	0.65

**Table 2:** Comparison of MRI diagnostic and pathological diagnosis results.

MRI	Pathological diagnosis		
	Malignant tumors (unit)	Benign tumors (unit)	Total
Malignant tumors (unit)	28 (35.00%)	13 (16.25%)	41
Benign tumors (unit)	7 (8.75%)	32 (40.00%)	39
Total	35	45	80
*χ* ^2^	1.02		
*P*	0.625		
Kappa	50.16%		

**Table 3:** Results of chest tumor detection at different sites.

		Pathological diagnosis		
MRI		Malignant tumors (unit)	Benign tumors (unit)	Total (unit)
Lung tumor	Benign (unit)	5 (6.25%)	3 (3.75%)	8
	Malignant (unit)	1 (1.25%)	6 (7.5%)	7
	Total (unit)	6	9	15
Mediastinal tumor	Positive (unit)	5 (6.25)	2 (2.5%)	7
	Benign (unit)	2 (2.5%)	7 (8.75%)	9
	Malignant (unit)	7	9	16
Chest wall tumor	Benign (unit)	5 (6.25)	3 (3.75%)	8
	Malignant (unit)	1 (1.25%)	4 (5%)	5
	Total (unit)	6	7	13
Esophageal tumors	Benign (unit)	6 (7.5%)	4 (5%)	10
	Malignant (unit)	2 (2.5%)	4 (5%)	6
	Total (unit)	8	8	16
Breast tumor	Benign (unit)	7 (8.75%)	1 (1.25%)	8
	Malignant (unit)	1 (1.25%)	11 (13.75%)	12
	Total (unit)	8	12	20

**Table 4:** Diagnostic efficacy of MRI in diagnosing chest tumors at different sites.

Site	Sensitivity	Specificity	Accuracy
Lung	83.33%	66.67%	73.33%
Mediastinum	71.43%	77.78%	75.00%
Chest wall	83.33%	57.14%	69.23%
Esophagus	75.00%	50.00%	62.50%
Mammary gland	87.50%	91.67%	90.00%

**Table 5:** Analysis of MRI imaging features of benign and malignant chest tumors.

Item	Feature	Malignant (unit) (*n* = 35)	Benign (unit) (*n* = 45)	*χ* ^2^	*P*
Morphology	Regular	2 (5.71%)	44 (97.78%)	73.7173	0.27
	Irregular	33 (94.29%)	1 (2.22%)		
Boundary	Distinct	1 (2.86%)	40 (88.89%)	63.5054	0.56
	Undistinct	33 (97.78%)	5 (11.11%)		
Invasion and lymph node metastasis	Yes	32 (91.43)	2 (4.44%)	70.43	0.09
	No	3 (8.57%)	43 (95.56)		

## Data Availability

The labeled dataset used to support the findings of this study are available from the corresponding author upon request.
